# Thyroid Dysfunction and Alopecia Areata: A Genetic Prediction Causality Analysis Study

This article has been retracted.

**DOI:** 10.1111/srt.70063

**Published:** 2024-09-27

**Authors:** Yue Zhao, Furong Guo, Mengyue Guo

**Affiliations:** ^1^ Department of Dermatology Heping Hospital Affiliated to Changzhi Medical College Changzhi China; ^2^ Changzhi Medical College Changzhi China

**Keywords:** alopecia areata, causal relationship, genetic evidence, Mendelian randomization, thyroid dysfunction

## Abstract

**Background:**

Observational studies have suggested a correlation between alopecia areata (AA) and thyroid dysfunction (TD). However, the causal relationship between AA and TD remains uncertain. The purpose of this study is to investigate the causal relationship between these two conditions. Understanding the potential causal relationship between AA and TD is valuable for elucidating the pathogenesis of AA and for designing innovative methods to prevent and treat AA and its related complications.

**Methods:**

All data for this two‐sample Mendelian randomization (MR) study were sourced from public databases. This study selected hypothyroidism, Hashimoto's thyroiditis, hyperthyroidism, subacute thyroiditis, and Graves' disease as exposure factors, with AA as the outcome variable. Data for hypothyroidism, Hashimoto's thyroiditis, hyperthyroidism, subacute thyroiditis, Graves' disease, and AA were obtained from related genome‐wide association studies (GWAS). Various MR analysis methods such as inverse variance weighted (IVW), MR‐Egger, and weighted median were utilized. Additionally, Cochrane's *Q* test was used to detect heterogeneity in MR results, and the MR‐Egger intercept test and MR pleiotropy residual sum and outlier (MR‐PRESSO) test were used to detect horizontal pleiotropy. A leave‐one‐out analysis was conducted to investigate the sensitivity of this association.

**Results:**

We found statistically significant genetic predictions of AA with hypothyroidism, Hashimoto's thyroiditis, and subacute thyroiditis (IVW OR = 1.4009815, 95% confidence interval [CI]: 1.1210399–1.750829; *p* = 0.003030698, OR = 1.396101, 95% CI: 1.030134–1.89208; *p* = 0.03144273, OR = 0.732702, 95% CI: 0.604812–0.887634; *p* = 0.001483368). Furthermore, tests for pleiotropy showed no evidence of pleiotropy, enhancing the credibility of the study results. Finally, the leave‐one‐out test demonstrated the stability and robustness of this association.

**Conclusion:**

This study provides new evidence of a potential genetic link between thyroid issues and AA. By employing the two‐sample MR method to eliminate confounding factors and reverse causation, unbiased results were obtained, confirming a causal relationship between hypothyroidism, Hashimoto's thyroiditis, subacute thyroiditis, and AA. This lays the foundation for further mechanistic studies and potential clinical applications. Future research should further explore the specific biological mechanisms between TD and the onset of AA.

## 1 Introduction

Alopecia areata (AA) is a common autoimmune skin disease, with a lifetime prevalence of about 2% worldwide [1]. It can occur at any age, but most cases are found in young people under 20 years old, with approximately 25%−50% of patients being younger than 20 years before the first onset [2]. The clinical presentation of AA primarily includes one or several round or oval bald patches with clear boundaries, where the skin surface is smooth and shows no obvious inflammatory response. In some cases, patients may experience rapid hair loss, leading to significant thinning of hair. Moreover, AA may be accompanied by changes in the nails, such as pitting or roughness on the nail surface. The course of AA is usually fluctuating, with possible spontaneous improvement or exacerbation of the condition [3, 4]. Genetic factors, environmental factors such as psychological stress, viral infections, and the use of certain medications are considered to be contributing factors to AA [5, 6]. AA not only affects the patient's appearance, but can also have a significant impact on their mental health, leading to decreased self‐esteem, social anxiety, and depression, among other psychological issues [7]. In some cases, AA may coexist with other autoimmune diseases, such as thyroid diseases [8]. Furthermore, recent research indicates a genetic causal relationship between asthma and AA, suggesting a possible link between AA and allergic diseases [9]. Due to the unpredictable course of AA, patients may experience multiple episodes of onset and remission, adding to the complexity of treatment and the psychological burden on the patient [10, 11].

Thyroid diseases, including hypothyroidism, Hashimoto's thyroiditis, hyperthyroidism, subacute thyroiditis, and Graves' disease, are common endocrine disorders worldwide. Thyroid hormones are essential for regulating metabolism, cardiovascular function, and the proliferation and differentiation of various cells [12]. Abnormal thyroid function can have a wide range of effects on the human body, including impacts on the health of skin and hair. Previous studies have shown that thyroid diseases are associated with various dermatological conditions, including AA, an immune‐mediated, non‐scarring folliculitis that leads to localized or generalized hair loss [8, 13]. Additionally, recent studies on the mutual effects of autoimmune diseases have also shown a genetic causal relationship between vitiligo and autoimmune thyroid diseases, further emphasizing the potential shared pathological mechanisms among these diseases [14].

Observational studies have identified a correlation between thyroid dysfunction (TD) and an increased incidence of AA [8, 15]. However, existing research often suffers from small sample sizes and limited data analysis methods, which restrict the generalizability and reliability of the results. Additionally, these studies have primarily focused on the direct effects of TD without adequately considering potential common risk factors, such as genetic background, environmental factors, and lifestyle, which could significantly influence the development of AA. This study aims to explore the relationship between thyroid issues and AA using a more systematic and comprehensive approach. Specifically, we employ genetic epidemiological methods, analyzing data from large population cohorts and applying statistical genetic tools, to uncover potential links between TD and the onset of AA. We hope this study will provide new insights into the interaction between thyroid diseases and AA and offer a scientific basis for developing potential treatment strategies.

## 2 Materials and Methods

### 2.1 Study Design and Data Sources

A two‐sample Mendelian randomization (MR) approach was used to explore the causal relationship between thyroid diseases (hypothyroidism, Hashimoto's thyroiditis, hyperthyroidism, subacute thyroiditis, Graves' disease) and AA. Compared to one‐sample MR, two‐sample MR utilizes separate and independent genome‐wide association studies (GWAS) data, making this method more effective and robust. In this study, thyroid diseases (hypothyroidism, Hashimoto's thyroiditis, hyperthyroidism, subacute thyroiditis, Graves' disease) were considered as exposure variables, and AA as the outcome variable. Single nucleotide polymorphisms (SNPs) were selected as instrumental variables (IVs) for further analysis (Figure 1). This study adheres to the three key assumptions of a two‐sample MR design: (1) all selected IVs are highly associated with the exposure (*p* < 5 × 10^−8^, *F*‐statistic > 10); (2) all selected IVs are independent of confounders between the exposure and outcome; (3) all selected IVs influence the outcome solely through the exposure and not via other pathways.

**FIGURE 1:** Three assumptions of the two‐sample MR study. MR indicates Mendelian randomization; SNP, single nucleotide polymorphism.

GWAS summary data for hypothyroidism, Hashimoto's thyroiditis, hyperthyroidism, and Graves' disease were obtained from specific literature PMID34594039 [16]. Hypothyroidism data included 30 155 cases and 379 986 controls. Hashimoto's thyroiditis data included 15 654 cases and 379 986 controls. Hyperthyroidism data included 3557 cases and 456 942 controls. Graves' disease data included 1678 cases and 456 942 controls. GWAS summary data for subacute thyroiditis were sourced from the Finnish Genome Consortium (https://r7.finngen.fi/), including 418 cases and 187 684 controls. All participants were of European descent, and informed consent was obtained from all participants. GWAS summary data for AA were also obtained from the Finnish Genome Consortium (https://r7.finngen.fi/), with the latest version including 289 cases and 211 139 controls.

**Table:** 

	GWAS Id	From	Population	Characteristics	Data	Number of SNPs
Graves' disease	ebi‐a‐GCST90018847	Literature:PMID34594039	European	Diagnosed as Graves' disease	458 620 (678 cases, 456 942 controls)	24 189 816
Hashimoto thyroiditis	ebi‐a‐GCST90018855	Literature:PMID34594040	European	Diagnosed as Hashimoto thyroiditis	395 640 (15 654 cases, 379 986 controls)	24 146 037
Hyperthyroidism	ebi‐a‐GCST90018860	Literature:PMID34594041	European	Diagnosed as hyperthyroidism	460 499 (3557 cases, 456 942 controls)	24 189 279
Hypothyroidism	ebi‐a‐GCST90018862	Literature:PMID34594042	European	Diagnosed as hypothyroidism	410 141 (30 155 cases, 379 986 controls)	24 138 872
Subacute thyroiditis	Finn‐b‐E4_THYROIDITSUBAC	Finnish Genome Consortium (https://r7.finngen.fi/)	European	Diagnosed as subacute thyroiditis	188 102 (418 cases, 187 684 controls)	16 380 373
Alopecia areata	finn‐b‐L12_ALOPECAREATA	Finnish Genome Consortium (https://r8.finngen.fi/)	European	Diagnosed as alopecia areata	211 428 (289 cases, 211 139 controls)	16 380 450

### 2.2 IV Selection

To conduct MR analysis, three assumptions must be adhered to: relevance, independence, and exclusion restriction. Therefore, all IVs used in further analysis must be rigorously selected. Initially, SNPs highly associated with the exposure (*p* < 5 × 10^−8^) were selected, excluding SNPs with *F*‐value < 10, ensuring significance and avoiding Weak IV bias. The formula for calculating *F*‐value is: *F* = *R* ^2^ × (*N*‐2)/(1‐*R* ^2^), where *R* ^2^ is the variance in the exposure explained by each IV. *R* ^2^ = 2 × EAF × (1‐EAF) × *β* ^2^, where *β* is the allele effect size and EAF is the effect allele frequency.

Secondly, due to potential biases from high linkage disequilibrium among selected SNPs, linkage disequilibrium pruning (*r*2 < 0.001, physical distance window = 10 000 kb) was performed to ensure IVs' independence. Thirdly, SNPs related to confounders and outcomes were excluded using PhenoScanner V2 software. Confounders in this study include hormone levels and endocrine changes, comorbidities, and medication use. This step ensures IVs influence the outcome solely through exposure.

### 2.3 Statistical Analysis

Statistical analysis was conducted using five different methods to test the genetic association between thyroid issues and AA: MR‐Egger regression, weighted median, inverse variance weighted (IVW), simple mode, and weighted mode. The IVW method, assuming all SNPs used in the analysis are valid, is expected to provide the most precise effect estimates. Hence, it is selected as the primary analysis method in this study. Statistical power was calculated on the website https://shiny.cnsgenomics.com/mRnd/, which allows for MR study statistical power calculations using the non‐centrality parameter method based on research by Brion et al. The power calculation requires the total *R* ^2^ value (variance) explained by each IV, with the *R* ^2^ calculation formula provided above. Some effective SNPs in Ensembles (https://useast.ensembl.org/index.html) corresponding genes in.

To ensure the reliability of the results, various tests were conducted. Cochrane's *Q* test was used to assess heterogeneity in the meta‐analysis. Additionally, funnel plots were used to detect heterogeneity based on their symmetry. The MR‐Egger intercept test and the MR pleiotropy residual sum and outliers (MR‐PRESSO) global test were used to detect pleiotropic effects. The MR‐PRESSO method can also detect outliers and provide effect estimates after excluding them. Finally, a leave‐one‐out sensitivity analysis was conducted to evaluate the stability of the results. By sequentially excluding SNPs and observing the effects of the remaining SNPs, it can be determined if a single SNP has a decisive impact on the overall association. All statistical analyses were completed using the TwoSampleMR package in R software (Version 4.2.0). A *p*‐value of < 0.05 was considered statistically significant.

## 3 Results

### 3.1 Selection of IVs

After excluding linkage disequilibrium, *F*‐value filtering, and adjusting for allele situations, 68 SNPs associated with hypothyroidism, 12 SNPs with Hashimoto's thyroiditis, 11 SNPs with hyperthyroidism, 4 SNPs with subacute thyroiditis, and 26 SNPs with Graves' disease were obtained. These SNPs served as the IVs for this study.

### 3.2 MR Analysis

Based on the IVW results, this study indicates a positive causal relationship between hypothyroidism, Hashimoto's thyroiditis, subacute thyroiditis, and AA. Hypothyroidism can increase the risk of AA (OR = 1.4009815, 95% confidence interval [CI]: 1.1210399–1.750829; *p* = 0.003030698 < 0.05), Hashimoto's thyroiditis can increase the risk of AA (OR = 1.396101, 95% CI: 1.030134–1.89208; *p* = 0.03144273 < 0.05), and subacute thyroiditis can increase the risk of AA (OR = 0.732702, 95% CI: 0.604812–0.887634; *p* = 0.001483368 < 0.05), as shown in Table 1. The genes corresponding to some effective SNPs are shown in Table 2.

**TABLE 1:** Effect of genetically determined TD on the risk of AA.

Exposure	MR methods	nSNP	*β*	SE	OR (95%CI)	*p*‐value
Graves' disease	MR Egger	26	0.2726	0.2628	1.313 (0.7847–2.198)	0.3099
	Weighted median	26	0.0764	0.1251	1.079 (0.8446–1.379)	0.5418
	IVW	26	0.0749	0.0890	1.078 (0.9053–1.283)	0.4002
	Simple mode	26	0.0228	0.2042	1.023 (0.6857–1.527)	0.9118
	Weighted mode	26	0.0767	0.1774	1.080 (0.7625–1.529)	0.6694
Hashimoto thyroiditis	MR Egger	12	0.6741	0.4408	1.962 (0.8271–4.655)	0.1572
	Weighted median	12	0.3622	0.2100	1.437 (0.9519–2.168)	0.0845
	IVW	12	0.3337	0.1551	1.396 (1.030–1.892)	0.0314
	Simple mode	12	0.3257	0.3199	1.385 (0.7398–2.593)	0.3306
	Weighted mode	12	0.3694	0.2454	1.447 (0.8945–2.341)	0.1603
Hyperthyroidism	MR Egger	11	−0.3865	0.3317	0.6794 (0.3546–1.302)	0.2739
	Weighted median	11	0.1048	0.1897	1.110 (0.7656–1.611)	0.5807
	IVW	11	−0.0045	0.1394	0.9955 (0.7575–1.308)	0.9742
	Simple mode	11	0.1982	0.3484	1.219 (0.6159–2.414)	0.5820
	Weighted mode	11	0.1490	0.2796	1.161 (0.671–2.008)	0.6056
Hypothyroidism	MR Egger	68	0.7002	0.2402	2.014 (1.258–3.225)	0.0049
	Weighted median	68	0.3460	0.1741	1.413 (1.005–1.988)	0.0469
	IVW	68	0.3372	0.1137	1.401 (1.121–1.751)	0.0030
	Simple mode	68	−0.0095	0.3644	0.9905 (0.4849–2.023)	0.9792
	Weighted mode	68	0.3468	0.1967	1.415 (0.9620–2.080)	0.0825
Subacute thyroiditis	MR Egger	4	−0.2081	0.2199	0.8121 (0.5277–1.250)	0.4439
	Weighted median	4	−0.2768	0.0943	0.7582 (0.6302–0.9121)	0.0033
	IVW	4	−0.3110	0.0979	0.7327 (0.6048–0.8876)	0.0015
	Simple mode	4	−0.5322	0.1723	0.5873 (0.4190–0.8233)	0.0538
	Weighted mode	4	−0.2185	0.1039	0.8037 (0.6556–0.9853)	0.1262

Abbreviations: AA, alopecia areata; IVW, Inverse variance weighted; MR, Mendelian randomization; TD, thyroid dysfunction.

**TABLE 2:** The genes corresponding to some effective SNPs.

SNP	Gene
rs10993994	MSMB, TSEN2xMSMB, PARG, TIMM23, MSMB
rs11065987	PTPN11, ATXN2, SH2B3, TRAFD1, ALDH2, BRAP, ALDH2, TRAFD1, SH2B3, SH2B3, ATXN2, CUX2, FAM109A, SH2B3, ATXN2, ACAD10, ALDH2, MAPKAPK5‐AS1, MAPKAPK5, ADAM1A, TMEM116, ERP29, NAA25, TRAFD1
rs1121980	FTO
rs11889341	STAT4
rs12726330	GBA
rs1333048	CDKN2A, CDKN2BxCDKN2A, CDKN2B
rs1421085	FTO, RPGRIP1L
rs16851483	RASA2
rs17782313	MC4R
rs203674	CFH
rs2074356	HECTD4, C12orf51, HECTD4, MYL2, CUX2, BRAP, ACAD10, ALDH2, MAPKAPK5, NAA25, TRAFD1, RPL6, OAS2, DTX1, C12orf51, ALDH2, FLJ30092
rs2245360	PAH
rs2287019	QPCTL, GIPR, QPCTL
rs2921053	CTA‐398F10.2
rs3184504	SH2B3, SH2B3, ATXN2, SH2B3, ATXN2, LOC100101246, BRAP, NAA25, C12orf51, PTPN11, ATXN2, SH2B3, CUX2, BRAP, ACAD10, SH2B3
rs3890745	TNFRSF14, MMEL1, TNFRSF14, MMEL1
rs4149057	SLCO1B1, NRxNR
rs6679677	PHTF1‐RSBN1, PTPN22, PHTF1, RSBN1, PHTF1, RSBN1, PTPN22, DCLRE1B, PTPN22, RSBN, PTPN22, PHTF1, PTPN22
rs73192661	LPP
rs11889341	STAT4
rs3184504	SH2B3, SH2B3, ATXN2, SH2B3, ATXN2, LOC100101246, BRAP, NAA25, C12orf51, PTPN11, ATXN2, SH2B3, CUX2, BRAP, ACAD10, SH2B3
rs6679677	PHTF1‐RSBN1, PTPN22, PHTF1, RSBN1, PHTF1, RSBN1, PTPN22, DCLRE1B, PTPN22, RSBN, PTPN22, PHTF1, PTPN22
rs73192661	LPP
rs78765971	VAV3

Abbreviation: SNPs, single nucleotide polymorphisms.

### 3.3 Sensitivity Analysis

The analysis results show that the MR‐Egger's egger‐intercept result has no statistically significant difference, indicating no horizontal pleiotropy in the results of this study; Cochran's *Q* test indicates that there are no statistically significant differences in the IVW results, and no heterogeneity is present, as shown in Table 3. MR‐Egger regression analysis showed that hypothyroidism, Hashimoto's thyroiditis, and subacute thyroiditis all had *p‐values* greater than 0.05, indicating that all SNPs included in the study were not affected by pleiotropy at the genetic level (Figure 2). The funnel plot showed that the scatter points representing each SNP were symmetrical, indicating no potential bias in the results (Figure 3). The leave‐one‐out test results showed that the IVW analysis results for the remaining SNPs were similar to the analysis results including all SNPs after sequentially excluding each SNP, with no significant impact on the assessment of causal associations by any single SNP, further confirming the stability of the results (Figure 4). Therefore, the MR results of this study are reliable.

**TABLE 3:** Heterogeneity test and horizontal pleiotropy test of TD‐associated SNPs.

Exposure	Horizontal pleiotropy		Heterogeneity	
	Egger‐intercept	*p*	Cochran's *Q*	*p*
Hypothyroidism	−0.042	0.092	69.88	0.381
Hashimoto thyroiditis	0.063	0.4277	10.42	0.404
Hyperthyroidism	0.094	0.236	8.293	0.600
Subacute thyroiditis	0.092	0.641	4.650	0.199
Graves' disease	0.045	0.432	22.79	0.590

Abbreviations: SNPs, single nucleotide polymorphisms; TD, thyroid dysfunction.

**FIGURE 2:** Scatter plots for this MR analyses of the causal relationship between TD and AA: (A)  hypothyroidism; (B) Hashimoto's thyroiditis; (C) subacute thyroiditis. AA indicates alopecia areata; MR, Mendelian randomization; TD, thyroid dysfunction.

**FIGURE 3:** Funnel plots for this MR analyses of the causal relationship between TD and AA: (A) hypothyroidism; (B) Hashimoto's thyroiditis; (C) subacute thyroiditis. AA indicates alopecia areata; MR, Mendelian randomization; TD, thyroid dysfunction.

**FIGURE 4:** MR leave‐one‐out sensitivity analyses of the causal relationship between TD and AA: (A) hypothyroidism; (B) Hashimoto's thyroiditis; (C) subacute thyroiditis. AA indicates alopecia areata; TD, thyroid dysfunction.

Moreover, the IVW results show that the association between the high genetic susceptibility to hyperthyroidism, Graves' disease, and a higher incidence of AA has no statistically significant difference.

## 4 Discussion

This study, based on GWAS data and employing the two‐sample MR method, has revealed a causal relationship between hypothyroidism, Hashimoto's thyroiditis, subacute thyroiditis, and AA, showing an increased risk of AA associated with hypothyroidism, Hashimoto's thyroiditis, and subacute thyroiditis. However, no causal relationship was found between hyperthyroidism, Graves' disease, and AA. The sensitivity analysis conducted using different MR models still presents robust results.

Increasing evidence suggests that TD can elevate the risk of developing AA [13, 15–17]. Specifically, in a study that included 89 patients with AA (with a median age of 40 years and a male‐to‐female ratio of 0.17), significant concurrent symptoms related to hypothyroidism were observed [18]. Furthermore, a prospective study utilizing data from the Nurses' Health Study (NHS), which included 63 692 women aged between 53 and 80, further confirmed this finding. The results indicate that individuals with a history of hypothyroidism showed a significantly increased risk of developing AA, manifested as a hazard ratio (HR) of 1.88, with a 95% CI extending from 1.30 to 2.71 [19].

Further research has revealed more complex interactions. For example, one study found that patients may be more susceptible to subacute thyroiditis, type 1 diabetes, chronic urticaria, or other autoimmune diseases before the onset of AA, suggesting that a broader autoimmune background may promote the development of AA [20]. Notably, the association between subacute thyroiditis and AA was confirmed in another retrospective case‐control study, where a certain proportion of AA patients were found to have subacute thyroiditis [21]. Research indicates that patients may be more susceptible to autoimmune diseases prior to the onset of AA, where the presence of Hashimoto's thyroiditis could potentially facilitate the development of AA [13, 21]. This correlation has been confirmed in one study, where a AA patient was found to have Hashimoto's thyroiditis, suggesting that a broader autoimmune background may promote the development of AA [22].

The relationship between AA and thyroid diseases, including hypothyroidism, Hashimoto's thyroiditis, and subacute thyroiditis, is complex, and the specific mechanisms by which these diseases increase the risk of AA are yet to be clarified. Studies have revealed that the neurophysiological disturbances associated with AA may be related to changes in monoamine neurotransmitter transmission, abnormal stress responses, and inflammatory reactions. An imbalance between dopamine and acetylcholine is considered a common final neuropathway for AA [23, 24]. Additionally, inflammation may induce a vulnerable physiological state, impairing brain function and increasing the permeability of the blood‐brain barrier, which could heighten susceptibility to endogenous toxins and pro‐inflammatory cytokines, leading to the development of AA [25].

Hypothyroidism, especially in the context of a deficiency in thyroid hormones, may be related to the development of AA through its impact on monoamine neurotransmitter transmission, abnormal stress responses, and inflammatory reactions [13]. As an autoimmune disease, Hashimoto's thyroiditis, as well as the inflammatory process involved in subacute thyroiditis, can lead to chronic inflammation and TD through immune attacks. The produced inflammatory cytokines (such as IFN‐γ, IL‐2, and TNF‐α) may indirectly affect distant hair follicle cells, inducing local inflammatory responses that interfere with the normal hair growth cycle and result in hair loss. Thyroid hormones are crucial for maintaining the normal physiological processes of skin and hair growth [26]. During this process, a decrease in thyroid hormone production could impact hair follicle proliferation and differentiation, causing the follicles to prematurely enter a resting phase, thereby triggering AA. Additionally, T cells, especially Th1 cells, play a key role in the immune attack on thyroid tissue and potentially on hair follicles, especially when the follicles express antigens similar to those of the thyroid tissue [27, 28].

Genetic studies have further revealed that the role of human leukocyte antigen (HLA) alleles in various autoimmune diseases has long been a focal point of research. These alleles can activate a large number of T lymphocytes and macrophages, destroying the immunity of hair follicles and leading to the occurrence of AA [29, 30].

Furthermore, the gene for cytotoxic T‐lymphocyte‐associated protein 4 (CTLA‐4), located on chromosome 2q33.2, encodes the CTLA‐4 protein. CTLA‐4 is homologous to CD28 and interacts with B7‐1/B7‐2 molecules on the surface of regulatory T cells (Treg cells), reducing the activation of T cells, and thereby inhibiting T cell proliferation and immune function [31]. Petukhova et al. [30] confirmed the association between the CTLA‐4 gene and the onset of AA through GWAS: High expression of the CTLA‐4 gene can inhibit the activity of Treg cells, thus participating in the occurrence of AA. Additionally, the reduction of the CTLA‐4 gene on T cells and polymorphisms in the CTLA‐4 gene can affect the expression and function of CD152, leading to abnormal activation and proliferation of T cells, which in turn triggers the onset of thyroid diseases [32, 33, 34]. Furthermore, the research conducted by Xu Wen and others provides compelling evidence showing that specific immunophenotypic traits such as CD62L‐CD86+ myeloid dendritic cells and TD CD4+%CD4+ T cells are associated with a protective effect against the risk of AA, while CD62L+ plasmacytoid dendritic cells and CD14‐CD16+ monocytes with HLA‐DR increase the risk of AA. These findings not only reveal the role of cytokines in the autoimmune process but also emphasize the critical function of these cells in regulating the immune privilege of hair follicles [35]. Moreover, factors such as infections, drugs, and psychological stress are associated with the occurrence of TD and AA [36, 37, 38]. These pieces of evidence suggest that both AA and TD are complex autoimmune diseases influenced by multiple genes and factors, and there is a close relationship between the two.

This study utilized the MR method to explore the relationship between thyroid diseases and AA, demonstrating the unique advantages of this method in revealing potential causal connections. Compared to traditional observational studies, MR, by using genetic variants as IVs, effectively reduces the impact of confounding factors, thereby enhancing the reliability of causal inferences.

Moreover, this study carefully selected genetic variants related to thyroid issues as IVs, based on previous research, to improve the precision of the MR analysis. However, the limitations of the study should also be fully recognized. First, the validity of the IVs is key to the success of an MR study. Any unknown confounding factors between the IVs and the outcome or associations with other risk factors could lead to biased analysis results. Second, although our study revealed potential associations between hypothyroidism, Hashimoto's thyroiditis, subacute thyroiditis, and AA, the specific biological mechanisms remain unclear and require further experimental research for exploration. Additionally, considering the impact of genetic heterogeneity and the representativeness of the data sources, our findings need to be validated in a broader population. This study provides preliminary evidence for a potential causal connection between thyroid issues and AA, but further research is necessary to verify the universality of these findings and uncover the specific underlying mechanisms.

## 5 Discussion

This study employed the MR method to explore the potential causal relationship between thyroid diseases and AA. Our findings indicate a significant association between hypothyroidism, Hashimoto's thyroiditis, subacute thyroiditis, and AA, suggesting a new perspective on the complex interplay between endocrine health and skin pathology. These discoveries not only provide new evidence for the relationship between TD and the pathogenesis of AA but also offer new directions for future research, especially in exploring potential treatments for AA.

## Conflicts of Interest

The authors declare no conflicts of interest.

## Data Availability

All data used in this study are publicly available from the respective GWAS databases. Specific URLs and access details are provided in the manuscript.
